# Diagnostic Value of IGFBP-2 in Predicting Preeclampsia before 20 Weeks of Pregnancy: A Prospective Nested Case-Control Study

**DOI:** 10.1155/2022/5075569

**Published:** 2022-09-28

**Authors:** Fei Gao, Jiaye Yin, Yan Long, Sufei Zhu, Zhenting Huang, Jielin Wang, Hao Zheng, Wen Wang, Lei Zheng

**Affiliations:** ^1^The First School of Clinical Medicine, Southern Medical University, Guangzhou 510515, China; ^2^Laboratory Medicine Center, Nanfang Hospital, Southern Medical University, Guangzhou 510515, China; ^3^Department of Laboratory, Guangzhou Women and Children's Medical Center, China

## Abstract

**Purpose:**

To identify novel biomarker insulin-like growth factor binding protein-2 (IGFBP-2) associated with preeclampsia (PE) before 20 weeks of gestation and to explore the predictive value of plasma IGFBP-2 in PE.

**Methods:**

A prospective nested case-control investigation involving 122 PE patients and 122 normal controls (NC) that were matched 1 : 1 in terms of age and week of pregnancy was carried out in Guangzhou Women and Children's Medical Center (Guangzhou, China, 2018030306) from April 2016 to December 2019. At 8 to 20 weeks, blood samples from the mother were taken. To calculate the correlations, univariate conditional logistic regression was employed.

**Results:**

Herein, 12 clinical indices were significantly different between the PE and NC groups (uric acid (UA), cystatin C (Cys C), aspartate aminotransferase (AST), glutamyl transpeptidase (*γ*-GT), total bilirubin (TB), prothrombin time (PT), red blood cell (RBC), hematocrit (HCT), red cell distribution width (RDW), platelets (PLT), mean platelet volume (MPV), and thrombocytocrit (PCT)). Compared with the NC group (36.79 ± 19.91 pg/mL), the expression level of IGFBP2 in the PE group (19.76 ± 19.40 pg/mL) before 20 weeks of pregnancy was significantly decreased (*P* < 0.01). Two high-risk factors were found to be significantly associated with PE independently of confounders: anemia 4.35 (2.20-8.45) (*P* < 0.01) and cesarean section history 8.25 (2.67-26.67) (*P* < 0.01). As a result of the univariate logistic regression analysis, the following three variables were included in the final logistic regression model.: *Y* = −18.841 − 0.085 × (IGFBP‐2) + 0.630 × (RDW) + 0.165 × (AST) + 0.863 × (MPV). In comparison to IGFBP-2 alone as an independent predictor of PE (AUC = 0.897, 95% CI 0.830–0.964), the model's discriminatory power was considerably higher (AUC = 0.953, 95% CI 0.911–0.995).

**Conclusion:**

Plasma IGFBP-2 before 20 weeks of pregnancy combined with high-risk factors and routine blood indexes has a high early predictive value for PE.

## 1. Introduction

Preeclampsia (PE) is a critical type of hypertensive disorder in pregnancy, manifested as persistently high blood pressure and proteinuria after 20 weeks of pregnancy, with an incidence of 3%-8% [1]. PE inhibits fetal intrauterine growth and affects several organs (including the liver, kidneys, lungs, and heart) as well as the nervous system of pregnant women. It also causes mortality, premature birth, and other problems. The programmed structural and functional changes caused by PE injury during pregnancy also elevate the risk of cardiovascular diseases after childbirth. Early screening of women at risk for PE can reduce the risk of preterm birth and early-onset preeclampsia by preventive measures, such as the use of aspirin and calcium [2].

Except for pregnancy termination, currently, there is no effective treatment that might underlie the risk of premature delivery. In clinical treatment, it is usually faced with the difficulty of deciding the maternal-fetal benefits [3–5]. Therefore, it is important to identify women who are at risk of PE in advance so that preventative and intervention strategies may be implemented. There are many biomarkers that have been suggested to predict PE. Presently, only a few effective clinical predictors have been identified for PE, resulting in a poor prognosis for the mother and perinatal infants and a sudden increase in the risk of death [6–8].

Several studies speculated that during the formation of PE placenta, extravillous trophoblast (EVT) suffers from decreased invasiveness and extravillous uterine spiral artery remodeling obstacle, resulting in shallow placenta implantation and poor placental vascular formation. In placental implantation, plasma proteins have a specific role as placental factors that induce endothelial dysfunction and a variety of other pathophysiological alterations linked to PE [9–11]. Due to the complexity and multifactorial nature of the disease, we employed antibody microarray technology to identify the crucial predictive proteins linked to PE.

Insulin-like growth factor binding protein 2 (IGFBP-2) belongs to the IGFBPs family, in which the content of IGFBP-2 is the second. IGFBP-2 was the first member found to be highly expressed in glioma, and it is associated with tumor differentiation, invasion, apoptosis, and angiogenesis [12, 13]. Placental microparticles may comprise fragments that are formed and released into the mother's blood circulation during pregnancy [14]. As a result, there is a lot of attention being paid to determining if there may be a difference in plasma IGFBP-2 levels between those with and without PE. The novel factor IGFBP-2 and previously known risk factors were incorporated in the current investigation to potentially increase the discriminatory performance of PE.

## 2. Methods

### 2.1. Study Design and Subjects

The research was based on an ongoing prospective study at the Guangzhou Women and Children's Medical Center (2018030306), Guangzhou, China, from April 2016 to December 2019. All subjects signed an informed consent, which was approved by the Ethics Committee of Guangzhou Women and Children's Medical Center. The samples were collected at enrollment, and the subjects followed up for up to 42 days postdelivery. Baseline demographic data and the mother's medical history and lifestyle information were collected.

In this nested case-control study, 5951 women were recruited during the discovery phase. PE occurred in 214 subjects, 122 of whom met all inclusion and exclusion criteria; the remaining patients were eliminated (Figure 1). These 122 PE-affected women were matched at a 1 : 1 ratio in terms of age, gestational week, and sample date to 122 controls who had uncomplicated pregnancies.

### 2.2. Diagnosis of PE

#### 2.2.1. Inclusion Criteria for Case Group

According to the expert consensus PE [15] in Guidelines for The Diagnosis and Treatment of Gestational Hypertension (2020), PE was defined as hypertension (systolic blood pressure ≥ 140 mmHg and/or diastolic blood pressure ≥ 90 mmHg) and proteinuria (urinary protein quantification > 0.3 g/24 h, or random urinary protein quantification ≥ 2+) emerging after 20 weeks of gestation. However, in the absence of proteinuria, hypertension should be accompanied by more than one of the following symptoms: (1) visual impairment, persistent headache, or other abnormalities of the central nervous system; (2) abnormal transaminase levels: elevated serum aspartate aminotransferase (AST) or alanine aminotransferase (ALT); (3) impaired renal function: urinary protein level > 2.0 g/24 h, or oliguria, or serum creatinine *level* > 106 *μ*mol/L; (4) hypoproteinemia with ascites, pleural effusion, or pericardial effusion; (5) platelet count continued to decrease to 100 × 10^9^ P/L; and (6) fetal growth restriction or oligohydramnios, intrauterine death, and placental abruption.

#### 2.2.2. Case Group Exclusion Criteria

Patients with a history of hypertension, kidney disease, or other conditions causing elevated blood pressure prior to the 20^th^ week of gestation were excluded. In addition, cases of primary lipid metabolism abnormalities, stillbirth, miscarriage, multiple pregnancies, fetal malformation, thyroid disease, gestational diabetes, and liver and kidney diseases were excluded [16].

#### 2.2.3. Inclusion Criteria for Normal Pregnancy

The pregnant woman gave birth to one full-term live fetus without any abnormalities.

### 2.3. Sample Collection

Women between 8 and 20 weeks of their pregnancies had their peripheral venous blood samples drawn, which were centrifuged at 3500 × g for 10 min at room temperature, and then promptly kept at -80°C. A total of 507 proteins of interest were found using a RayBio Label-based Human Antibody Microarray (catalog # AAH-BLG-1; RayBiotech, Norcross, GA, USA). Assays were carried out as per the manufacturer's instructions. Because of the challenges in collecting early pregnancy plasma samples from women with PE, only IGFBP-2 levels were examined as they showed a high fold-change among the downregulated proteins in the protein microarray. IGFBP-2 is also essential in trophoblastic immune privilege and trophoblast invasion in the early stages of pregnancy. IGFBP-2 plasma concentrations were measured by ELISA kit (Bes11047H, BersinBio, Guangzhou, China).

### 2.4. Data Collection

On the basis of a literature review and clinical expertise, the potential risk factors were chosen. Medical records were used to collect the data. Sociodemographic characteristics (maternal age, gestational age, body mass index (BMI), ethnicity, and place of birth), pregnancy history, past medical history, family history (gestational diabetes mellitus and hypertension), and adverse perinatal outcomes (scar uterus, oligohydramnios, premature rupture of membranes, postpartum hemorrhage, premature delivery, and low birth weight) were the included variables. Routine blood indices (blood routine, coagulation function, liver function, and kidney function) before 20 weeks of gestation were collected and analyzed.

### 2.5. Statistical Analysis

Data analysis was carried out using SPSS 26.0 software. The normal-distribution measurement results were expressed as mean ± standard deviation (SD), and an independent sample test was employed to compare the variables across groups. Median (interquartile spacing) (*M* (P25, P75)) was used for skewed distribution. Wilcoxon rank-sum test or Mann–Whitney *U* test was utilized to compare the variables across groups. For the correlation analyses, Spearman correlation analysis was utilized. Single factor analysis was used for screening significant risk factors, and multivariate logistic regression analysis was utilized for determining the prediction model of PE. The receiver operating characteristic (ROC) curve was drawn by using a stepwise logistic regression model to determine the sensitivity, specificity, negative/positive likelihood ratio, and other indicators, and the predictive value of indicators was evaluated by the area under the curve (AUC) value. *P* < 0.05 was taken as significant.

## 3. Results

### 3.1. Demographical Data

In total, 244 pregnant women, 122 of whom were in the PE group and 122 of whom were in the normal pregnancy group, were enrolled in this study. Before 20 weeks of gestation, the BMI level of the PE group was higher in comparison to that of the normal pregnancy group (*P* < 0.05); however, there were no significant differences detected in the race, nationality, age, and gestational age between the two groups (*P* > 0.05). The results were as follows: in the PE group, the changes in blood cell system, the red blood cell count, hematocrit, red blood cell distribution width, mean platelet volume and specific platelet volume, serum uric acid and cystatin C, serum aspartate aminotransferase, glutamyl transpeptidase, and total bilirubin levels in the liver function test, and prothrombin time were higher in comparison to those in the normal group (*P* < 0.05), while platelet count was lower than the normal group. No statistical difference was observed in the other items (Table 1).

### 3.2. Analysis of High-Risk Factors and Adverse Outcomes

Univariate analysis showed that history of anemia and cesarean section were statistically significant in the PE group (*P* < 0.05). The relative risk odds ratio (OR) (95% confidence interval (CI)) values of anemia and cesarean section history are 4.35 (2.20-8.45) and 8.25 (2.67-26.67), respectively. The probability of high risk of placenta accreta, scar uterus, oligohydramnios, abnormal placenta, and low birth weight in the PE group was remarkably higher in comparison to that in the normal pregnancy group (*P* < 0.05). The relative risk OR (95% CI) of high risk of placenta accreta, scar uterus, oligohydramnios, and placental abnormality in pregnancy was 2.33 (1.18-26.67), 9.71 (2.93-31.19), 25.16 (4.41-263.70), and 3.82 (1.28-10.89), respectively. And then, the relative risk OR (95% CI) of low birth weight was 49.08(8.21-505.90). On the other hand, there was no significant difference observed between the PE group and normal groups in pregnancy times and history of spontaneous abortion (*P* > 0.05) (Table 2).

### 3.3. Correlation between Plasma IGFBP-2 Expression Level and Routine Laboratory Indicators

The plasma IGFBP-2 expression level before 20 weeks of pregnancy was detected by enzyme-linked immunosorbent assay (ELISA). A total of 100 pregnant women (50 in the NC group and 50 in the PE group) were detected before 20 weeks of pregnancy. As a result, before 20 weeks of pregnancy, the level of IGFBP-2 in the PE group (19.76 ± 19.40 pg/mL) was substantially lower in comparison to that in the normal group (32.59 ± 17.90 pg/mL) (*P* < 0.01) (Figure 2).

Spearman's correlation analysis was carried out to assess the expression level of plasma IGFBP-2 before 20 weeks of pregnancy in the PE group and routine laboratory indicators. The outcomes demonstrated that the plasma IGFBP-2 expression level before 20 weeks of pregnancy was negatively correlated with AST, RBC, RDW, and MPV (*r* = −0.34, -0.25, -0.31, -0.30; *P* < 0.01) in PE; however, there was no statistically significant correlation with other indicators (Table 3).

### 3.4. Efficacy of the Predictive Model

The statistically significant high-risk factors and clinical indicators were included in the regression analysis, and the stepwise logistic regression analysis was adopted. Finally, the regression analysis model was obtained: *Y* = −18.841 − 0.085 × (IGF BP‐2) + 0.630 × (RDW) + 0.165 × (AST) + 0.863 × (MPV) (Table 4).

Using ROC analysis of IGFBP-2 levels, the discriminatory capacity of IGFBP-2 and the clinical factors related to PE were evaluated (Figure 3). Using IGFBP-2 as a single predictor, the AUC was 0.897 (95% CI 0.830–0.964) with 86.0% sensitivity and 84.0% specificity. Subsequently, the AUC increased to 0.953 (95% CI 0.911–0.995) with 94.0% sensitivity and 88.0% specificity when clinical factors for PE were entered into the logistic model based on the optimal cutoff point (Table 5).

## 4. Discussion

We found plasma IGFBP-2 levels before 20 weeks of gestation in this nested case-control research from a cohort of Chinese pregnant women to be prospectively linked to the risk of PE. In the Chinese population, the level of IGFBP-2 is predicted for 89.7% of PE cases. The combination of improved the detection rate of PE to 95.3%. The inclusion of IGFBP-2 improved the PE prediction beyond conventional risk factors and clinical markers. To our knowledge, this is the first study to investigate the predictive value of IGFBP-2 on PE in the Chinese population, which provides a novel perspective for the prediction of PE.

Maternal markers, ultrasound markers, and biomarkers including PIGF, sFlt-1, and PAPP-A have all been employed for PE prediction [6–8]. Based on several studies on the early markers for PE recognition, several multiparameter algorithms have been developed. In summary, although a large number of markers and algorithms have been studied, a reliable PE prediction model has not been developed. Presently, there is no clinically significant screening test available for the prediction of PE development. The abnormal vascular remodeling of the spiral arteries in the uterus, resulting in superficial implantation of the placenta, might be the pathogenesis of PE. With the use of maternal trophoblast invasion factors like IGFBP-2, this condition can be used to predict PE. IGFBP-2 levels in the blood of pregnant women who later developed PE were shown to be lower in earlier studies. Recent studies consistently show that in early pregnancy (before 20 weeks gestation), the plasma level of IGFBP-2 in the PE group was substantially lower in comparison to that in the control group (Figure 2). In addition, IGFBP-2 can regulate the inflammatory response, apoptosis, differentiation invasion, and angiogenesis through multiple signaling pathways such as the Ras-MAPK pathway, PI-3K/AKT pathway, JNK pathway, P53, PTEN, and Wnt/*β*-catenin molecules [17–23]. In this study, it was found for the first time that the plasma IGFBP-2 level decreased before 20 weeks of pregnancy in the PE group, which inhibited the invasion of EVT and caused PE. Simultaneously, the expression level of IGFBP-2 was negatively correlated with AST, RBC, RDW, and MPV (Table 3).

Several studies reported that social, nutritional, blood, inflammation, immune, genetic, and other factors would affect the occurrence of PE [24, 25]. In this study, the red blood cell count, red blood cell distribution width, and prothrombin time in the PE group were higher in comparison to those in the normal group. Reportedly, the increase in RBC distribution width is due to the influence of inflammatory factors on RBC production and deformation ability [26, 27]. This study found that red blood cell count in the PE group increased significantly in early pregnancy, which might be due to the compensatory response caused by microcirculation ischemia and hypoxia in the body. An increased number of red blood cells in pregnant women, insufficient blood volume, and blood viscosity also lead to microthrombosis in PE pregnant women, thereby aggravating disorders related to blood circulation [28]. The liver and kidney function indicators (glutamyl transpeptidase, aspartate transferase, creatinine, and cystatin C) in the PE group were increased, which was consistent with the study by van der Tuuk et al. [29]. The pregnant women with PE had specific organ damage before they showed significant hypertension and proteinuria in the early pregnancy. Due to individual differences and the compensatory phase of organ damage, imaging and test indicators may still be within the normal range and not detected easily [30–33]. The combined assessment of risk factors and blood indicators in early pregnancy may play an important role in identifying high-risk groups for PE.

In the current study, anemia and cesarean section history were also found to be different between the PE and NC groups, consistent with previous studies. The highest relative risk in our study was the history of cesarean section. This procedure caused scar uterus, which was prone to dysplasia of the placental decidua, aggravating the symptoms of placental ischemia and hypoxia and leading to spasmodic contraction of small arteries and inducing PE. Placental tissue changes caused by anemia during pregnancy are characterized by dysregulation of the pregnancy-placental-fetal system and placental tissue ischemia in response to hypoxia [34]. PE can cause multiple complications and adverse pregnancy outcomes for both mothers and babies. In this study, the PE group had an increased risk of Down's syndrome, scar uterus, oligohydramnios, and placental abnormalities (*P* < 0.05). In addition, the proportion of low-birth-weight infants in the PE group was considerably higher in comparison to that in the NC group (*P* < 0.01).

In addition, in the present study, when IGFBP-2 was incorporated into the logistic model as a novel factor, the AUC was 0.897 (95% CI 0.830–0.964) with 86.0% sensitivity and 84.0% specificity, and the model had a high discriminatory performance for PE (Table 5). This indicates that plasma IGFBP-2 before 20 weeks of pregnancy may have a predictive effect on PE. In comparison to the levels of angiogenic factors or placental hormones in the first trimester, our model has excellent discriminatory power.

According to a prospective study by Skråstad et al., the AUC for placental growth factor was 0.63 [35]. Abdelaziz et al. reported an AUC of 0.57 for soluble endoglin [36]. In a longitudinal study by Akolekar et al., the AUC values for placental protein 13 and pregnancy-associated plasma protein A were 0.82 and 0.87, respectively. According to the ROC curve, IGFBP-2 is a good biomarker for predicting the occurrence of preeclampsia in early pregnancy. In this study, the prediction and diagnosis rates of preeclampsia were improved to a certain extent by combining high-risk factors (anemia, cesarean section history), blood routine, coagulation routine, and liver and kidney function. The obtained logistic regression model combined with clinical risk factors prediction: *Y* = −18.841 − 0.085 × (IGFBP‐2) + 0.630 × (RDW) + 0.165 × (AST) + 0.863 × MPV.

Nevertheless, the present study has some limitations. Although many pregnant women were enrolled in our cohort, the number of women who developed PE was insufficient, thus limiting the accuracy of our relative risk estimates. In addition, all women in our investigation were from the same province, which might lead to a bias in the outcomes that should be validated by a prospective multicenter clinical study. Since the study's controls excluded participants who had abnormal results, there may have been a bias with overestimation of discriminatory power. Herein, we validated only IGFBP-2 levels because it showed the higher-fold change among the downregulated proteins in the protein microarray. To further enhance the discriminatory performance, we will substantiate the expression of the other 24 differentially expressed proteins in subsequent research.

In conclusion, plasma IGFBP-2 before 20 weeks of pregnancy combined with high-risk factors and routine blood indices has a high early predictive value for preeclampsia.

## Figures and Tables

**Figure 1:** Flow diagram of study design.

**Figure 2:** Comparison of IGFBP-2 levels between the PE group and NC groups.

**Figure 3:** ROC curve of single and combined IGFBP-2 in predicting preeclampsia.

**Table 1:** Clinical data of the PE group and control groups.

Variables	PE (*n* = 122)	NC (*n* = 122)	*P*
Han, *n* (%)	118 (96.72)	119 (97.54)	0.99
Guangdong nationality, *n* (%)	90 (73.77)	89 (72.95)	0.99
Age (years)	32.37 ± 4.82	32.48 ± 4.50	0.87
Gestational weeks	16.75 ± 2.56	17.18 ± 2.27	0.19
BMI (kg/m^2^)	26.21 ± 5.17	24.83 ± 3.63	0.01
*Renal function indexes*			
UA (*μ*mol/L)	271.0 (228.0, 310.5)	217.5 (191.0, 248.8))	<0.01
Cr (*μ*mol/L)	43.0 (38.0, 46.0)	42.0 (37.0, 47.0)	0.73
Urea (mmol/L)	2.75 (2.19, 3.23)	2.82 (2.44, 3.38)	0.20
Cys C (mg/L)	0.59 (0.49, 0.71)	0.55 (0.45, 0.62)	<0.01
*Liver function indexes*			
ALT (U/L)	16.00 (11.00, 26.00)	16.00 (12.00, 26.25)	0.30
AST (U/L)	21.00 (18.00, 26.00)	17.00 (14.00, 21.00)	<0.01
*γ*-GT (U/L)	12.50 (10.00, 17.00)	11.00 (8.00, 14.00)	<0.01
TB (*μ*mol/L)	8.90 (7.55, 10.95)	7.00 (5.80, 9.25)	<0.01
*Blood coagulation indexes*			
PT (s)	12.10 (11.70, 12.40)	11.80 (11.50, 12.30)	<0.01
APTT (s)	33.10 (31.20, 34.55)	32.40 (30.38, 34.83)	0.28
TT (s)	16.00 (15.45, 16.55)	15.80 (15.20, 16.30)	0.34
Fib (g/L)	4.69 ± 0.89	4.66 ± 0.70	0.82
*Blood routine indexes*			
RBC (10^12^/L)	4.09 (3.77, 4.45)	3.85 (3.64, 4.11)	<0.01
HB (g/L)	119.9 ± 11.39	118.8 ± 9.70	0.36
HCT (%)	36.30 (34.00, 38.53)	35.00 (33.10, 36.70)	<0.01
RDW (%)	16.20 (14.53, 16.80)	13.05 (11.50, 15.00)	<0.01
PLT (10^9^/L)	224.8 ± 51.15	253.0 ± 55.31	<0.01
MPV (fL)	10.75 (9.90, 11.40)	8.10 (7.70, 9.03)	<0.01
PCT (%)	0.24 ± 0.05	0.21 ± 0.05	<0.01

**Table 2:** Analysis of high-risk factors and adverse outcomes between the NC group and PE groups.

	PE (*n* = 122)	NC (*n* = 122)	OR (95% CI)	*P*
*High-risk factors*				
Anemia, *n* (%)	44 (36.07)	14 (11.48)	4.35 (2.20-8.45)	<0.01
History of diabetes	0 (0)	0 (0)	N	N
History of hypertension	1 (0.8)	0 (0)	N	0.99
Gravidity = 1, *n* (%)	39 (31.97)	37 (30.33)	1.08 (0.63-1.85)	0.78
Gravidity ≥ 3, *n* (%)	49 (40.16)	39 (31.97)	1.43 (0.84-2.38)	0.18
History of preterm birth, *n* (%)	1 (0.8)	1 (0.8)	N	N
Spontaneous abortion ≥ 2, *n* (%)	11 (9.02)	7 (5.74)	1.63 (0.61-4.19)	0.33
Cesarean delivery, *n* (%)	21 (17.21)	3 (2.46)	8.25 (2.67-26.67)	<0.01
Stillbirths, *n* (%)	1 (0.8)	0 (0)	N	0.99
*Adverse pregnancy and perinatal outcomes*				
High risk of Down's screening, *n* (%)	30 (24.60)	15 (12.30)	2.33 (1.18-26.67)	0.01
Scar uterus, *n* (%)	24 (19.67)	3 (2.46)	9.71 (2.93-31.19)	<0.01
Oligohydramnios, *n* (%)	21 (17.21)	1 (0.8)	25.16 (4.41-263.70)	<0.01
Premature rupture of membranes, *n* (%)	25 (20.49)	15 (12.30)	1.84 (0.94-3.66)	0.08
Placenta abnormality, *n* (%)	14 (11.48)	4 (3.28)	3.82 (1.28-10.89)	0.03
Postpartum hemorrhage, *n* (%)	1 (0.8)	4 (3.28)	0.24 (0.02-1.51)	0.37
Preterm birth, *n* (%)	3 (2.46)	0 (0)	N	0.25
Fetal weight (<2500 g)	35 (28.69)	1 (0.8)	49.08 (8.21-505.90)	<0.01

N: defy calculation.

**Table 3:** Correlation analysis between the plasma IGFBP-2 expression level and clinical index.

	*r*	*P*
UA (*μ*mol/L)	-0.18	0.07
CysC (mg/L)	-0.05	0.62
AST (U/L)	-0.34	<0.01
*γ*-GT (U/L)	-0.13	0.18
TB (*μ*mol/L)	-0.03	0.79
PT (s)	-0.13	0.19
RBC (10^12^/L)	-0.25	<0.01
HCT (%)	-0.14	0.18
RDW (%)	-0.31	<0.01
PLT (10^9^/L)	-0.11	0.25
MPV (fL)	-0.30	<0.01
PCT (%)	0.012	0.91

**Table 4:** Logistic regression analysis of risk factors for PE.

Risk factor	*B*	SE	Wald	*P*	OR (95% CI)
IGFBP-2	-0.085	0.034	6.141	0.013	0.918 (0.858, 0.982)
RDW	0.630	0.194	10.590	0.001	1.878 (1.285, 2.745)
AST	0.165	0.056	8.756	0.003	1.179 (1.057, 1.315)
MPV	0.863	0.234	13.566	0.001	2.371 (1.498, 3.753)

**Table 5:** Evaluation of AUC and related parameters by IGFBP-2 and joint index.

Variable	AUC ± SD	*P*	(95% CI)
IGFBP-2 prediction probability	0.897 ± 0.034	<0.01	0.830-0.964
Combined prediction probability	0.953 ± 0.021	<0.01	0.911-0.995

## Data Availability

The data used to support the findings of this study are included within the article.
